The article "Double Positive CD4CD8 αβ T Cells: A New Tumor-Reactive Population in Human Melanomas" was published in 2010. Journal: PLoS One.

# Double Positive CD4CD8 αβ T Cells: A New Tumor-Reactive Population in Human Melanomas

**DOI:** 10.1371/journal.pone.0008437

**Published:** 2010-01-05

**Authors:** Juliette Desfrançois, Agnès Moreau-Aubry, Virginie Vignard, Yann Godet, Amir Khammari, Brigitte Dréno, Francine Jotereau, Nadine Gervois

**Affiliations:** 1 UMR INSERM, U892, Nantes, France; 2 Université de Nantes, Faculté des Sciences, Nantes, France; 3 Unit of Skin Cancer, Centre Hospitalier Universitaire de Nantes, Nantes, France; 4 GMP Unit of Cellular Therapy, Centre Hospitalier Universitaire de Nantes, Nantes, France; Cedars-Sinai Medical Center and University of California Los Angeles, United States of America

## Abstract

**Background:**

Double positive (DP) CD4CD8 Tαβ cells have been reported in normal individuals as well as in different pathological conditions including inflammatory diseases, viral infections and cancer, but their function remains to be elucidated. We recently reported the increased frequency of DP Tαβ cells in human breast pleural effusions. This manuscript addresses the question of the existence and above all the role of this non-conventional DP sub-population among tumor associated lymphocytes in melanomas.

**Methodology/Principal Findings:**

We analyzed the intratumoral cell infiltrate in solid metastasis (n = 6) and tumor invaded lymph nodes (n = 26) samples from melanomas patients by multiparametric cytometry. Here we documented for the first time significant increased frequency of DP T cells in about 60% of melanoma tumors compared to blood samples. Interestingly, a high proportion of these cells produced TNF-α in response to autologous melanoma cell lines. Besides, they are characterized by a unique cytokine profile corresponding to higher secretion of IL-13, IL-4 and IL-5 than simple positive T cells. In deep analysis, we derived a representative tumor-reactive DP T cell clone from a melanoma patient's invaded lymph node. This clone was restricted by HLA-A*2402 and recognized both autologous and allogeneic tumor cells of various origins as well as normal cells, suggesting that the target antigen was a ubiquitous self antigen. However, this DP T cell clone failed to kill HLA-A*2402 EBV-transformed B cells, probably due to the constitutive expression of immunoproteasome by these cells.

**Conclusions/Significance:**

In conclusion, we can postulate that, according to their broad tumor reactivity and to their original cytokine profile, the tumor associated DP T cells could participate in immune responses to tumors *in vivo*. Therefore, the presence of these cells and their role will be crucial to address in cancer patients, especially in the context of immunotherapies.

## Introduction

In the last 20 years, T lymphocytes reactive to antigens expressed by tumor cells have been shown to modulate cancer development in animal models and human cancer patients [1], [2]. Thus, much effort has been devoted to the development of immunotherapeutic strategies aimed at inducing cancer regression by enhancing antigen T cell responses [3]. Active (cancer vaccines) and adoptive (infusion of tumor-reactive cells) immunotherapies tested in clinical trials have produced tumor regression, proving that the immune system can be harnessed to kill tumor cells in cancer patients [4]–[6]. However, the efficacy of such strategies remains quite limited and needs to be improved. It is now clear that most cancer patients do not develop a satisfactory immunological anti-tumor response due to the existence of tumor-specific immune evasion strategies. Until now, several mechanisms have been described including alteration of MHC class I and tumor antigen expression by tumor cells, secretion of immunosuppressive soluble factors either by tumor cells or infiltrating T cells or both [7]. Recent studies have demonstrated that one of the major mechanisms responsible for the downregulation of T-cell responses against tumors is the presence of several types of suppressor cells within the tumor. These suppressor cells include the now-classical T reg cells and the more recently described type II NKT cells [8], [9]. We hypothesized that insights into these mechanisms could be gained from the study of T cell infiltration in tumor and especially of unconventional and regulator cell populations.

We previously reported in breast cancer patients that, in addition to conventional CD4^+^ and CD8^+^ αβ T cells, individual tumors and most pleural effusions contained significant fractions of unconventional double positive (DP) CD4^+^CD8^+^ αβ T cells [10]. DP T cells have been reported as a small population in the peripheral blood of healthy individuals, increasing with age [11]. Furthermore, these cells may be increased in patients with autoimmune diseases and viral infections [12]–[14]. They have also been reported in cutaneous T-cell lymphoma and in nodular lymphocyte predominant Hodgkin lymphoma [15], [16]. Our earlier study reported that the breast tumor associated DP T cells displayed the phenotype and cytotoxic potential of effector/memory activated CD8^+^ T cells but differed essentially from these cells by a high production of IL-4, IL-5 and IL-13 [10]. The increased frequency of DP T cells in advanced breast cancer as well as their high lytic potential and original cytokine profile suggest that these cells might play a significant role in regulating immune responses to human cancer. However, these breast cancer associated DP T cells were not characterized with respect to anti-tumor reactivity due to the difficulty of establish *in vitro* autologous tumor cell lines in this model.

This led us to perform the current study in human melanomas to determine the presence of DP T cells and their anti-tumor reactivity. Examination of T cell subsets in metastasis and invaded lymph nodes from melanoma patients revealed a significantly increased proportion of DP T cells including autologous tumor-reactive cells. We successfully isolated one autologous tumor-specific DP T cell clone which has been characterized in terms of functional properties and antigen specificity.

## Results

### Enhanced Frequencies of Tumor-Reactive DP T Cells in Melanomas

We analyzed the intratumoral cell infiltrate in solid metastasis (n = 10) and tumor invaded lymph nodes (n = 26) samples from melanomas patients by flow cytometry. To get a sufficient number of TAL (Tumor Associated Lymphocytes) for extensive characterization, a single expansion of these cells was done using PHA and feeder cells. For comparison purposes, a similar phenotypic analysis was performed on fresh PBMC derived from healthy donors (n = 11) and from stage III melanoma patients (n = 6). As expected, most tumor infiltrating populations obtained after in vitro expansion consisted of a majority of CD3 positive T cells often exceeding 98%. As shown on Table 1, frequencies of SP CD4^+^ T cells were similar in PBMC and TAL whereas the CD8^+^ subset was statistically higher in tumors, especially in invaded lymph nodes (P<0.001). Significant fractions of DP T cells were observed in about 60% of melanoma cases and represented 4.3% of ILNL (Invaded Lymph Node Lymphocytes) and 9.5% of TIL (Tumor Infiltrating Lymphocytes). In contrast, this population did not exceed 1% in PBL from melanoma patients as well as in PBL from healthy donors. The prevalence of DP T cells in metastatic tumors was significantly higher (P<0.05) than in invaded lymph nodes and still higher (P<0.01) than in normal or patients blood.

**Table 1:** Distribution of T cells subsets based on CD3, CD4, CD8 amongst melanoma patients PBMC and tumor associated lymphocytes and healthy donor PBMC.

	FREQUENCY			
Cell origin	CD3^+^	CD4^+^	CD8^+^	CD4^+^CD8^+^
**PBMC**				
*healthy donors (n = 11)*	70,5+/−6,3	46+/−10	9.5+/−9	0.9+/−0.6
*melanoma patients (n = 6)*	68,5+/−7,1	51.1+/−6	14.9+/−3	0.6+/−0.2
**Melanoma Associated Lymphocytes**				
*ILNL (n = 30)*	99,9+/−0,2*	31.1+/−26	54.2+/−25***	**4.2**+/−5.6
*TIL (n = 10)*	98,4+/−9,1*	35,3+/−26	50,3+/−26**	**9,5**+/−8,3**

Results are expressed as median fraction of cells expressing the marker(s) +/− SD among total cells. Significant differences were evaluated by comparison with similar cell fractions among melanoma cancer patient PBMC using the Tukey-Kramer's test. *P<0.05, **P<0.01, ***P<0.001.

In order to evaluate their repertoire diversity, the pattern of TCR Vβ usage of four DP T cells populations was determined with a panel of 24 anti-Vβ antibodies representing the most frequently expressed Vβ chains within a normal repertoire (Figure 1A). We showed that despite the strong dominance of DP lymphocytes expressing one particular Vβ chain (2, 11 or 13.2) in two out of four melanoma invaded lymph nodes (M134 and the M314), the repertoire analysis of these DP T cells populations was relatively diverse and did not reveal any recurrence of a particular Vβ usage.

**Figure 1:** Analysis of polyclonal DP T cells in melanoma: repertoire diversity and autologous-tumor reactivity. A/ Repertoire diversity of DP T cells populations in tumors from four melanoma patients was assessed by labeling with 24 anti-Vβ mAbs. Insets indicate the percentage of the specific population characterized with this panel. B/ Percentage of TNF-producing cells in the SP CD8 and DP sub-populations in response to the autologous melanoma cell line. The autologous tumor cells lines were established from metastatic lymph nodes of 21 melanoma patients and were tested after two at four weeks of culture initiation. 10^6^ ILNL and 2×10^6^ melanoma cells were incubated for 6 h in the presence of Brefeldin A, stained with CD4 and CD8 mAbs, fixed, and stained with anti-TNF Ab in a permeabilization buffer. 10^5^ cells were then analyzed by flow cytometry.

We then analyzed by flow cytometry the cytokine secretion profile of DP T cells derived from solid tumors (n = 4) and from invaded lymph node (n = 1) compared with SP CD4^+^ and CD8^+^ T cells. Since results did not differ as a function of the TAL origin, data were pooled in Table 2.

**Table 2:** Comparison of cytokine production capacities of DP T cells with that of SP subpopulations by FACS analysis.

		CD4	CD8	DP
**CYTOKINE PRODUCTION**	***TNF-α***	63+/−12	79+/−12	82+/−10
	***IFN-γ***	32+/−16	49+/−29	46+/−13
	***IL-2***	28+/−11	35+/−17	48+/−14
	***IL-4***	22+/−10	23+/−5	40+/−11*
	***IL-5***	2+/−1	5+/−2	21+/−7***
	***IL-13***	28+/−10	35+/−11	75+/−12***
	***GM-CSF***	48+/−22	53+/−22	74+/−11

Data are expressed as mean % of intracellular cytokine secreting cells in response to anti-CD3 stimulation (n = 5). Significance increase of cytokines production by DP T cells was evaluated by Tukey-Kramer's test. *P<0.05,***P<0.001. No cytokine production was observed by unstimulated subpopulations.

Mean fractions of TAL subsets secreting TNF-α and IFN-γ upon stimulation by anti-CD3 were similar. In contrast, the percentages of IL-2, IL-4, IL-5, IL-13 and GM-CSF secreting cells were higher among DP T cells than among SP T cells. This was especially clear for IL-4 (P<0.05), IL-5 and IL-13 (P<0.001) with respectively a mean of 40%, 21% and 75% of DP T cells secreting these cytokines whereas these percentages did not exceed 23%, 5% and 35% in the SP subpopulations.

To evaluate the tumor reactivity of this new DP population, we derived melanoma cell lines from tumor samples. The tumor reactivity was evaluated by the percentages of SP CD8 and DP T cells producing TNF-α in response to autologous melanoma cells. Twenty one populations of short term culture TAL could be analyzed and as shown on Figure 1B, more than fifty of these contained a significant fraction (>2%) of autologous melanoma reactive T cells among the DP population as well as among the SP CD8 population. Moreover, the mean percentage of cells producing TNF-α in response to autologous melanoma was superior in DP T cells than in SP CD8 T cells (14.7% versus 4.7%).

### DP T Cell Clone Selection and Characterization

To facilitate the characterization of the DP T cell population, we derived tumor-reactive T cell clone from the M314 ILNL population containing 14% of DP T cells among which about 60% expressed the Vβ13.2 TCR and were reactive against the autologous melanoma cell line (Figure 2A). The Vβ13.2 expressing T cells were sorted by FACS and sequenced for CDR3 (data not shown), that allow us to conclude that this Vβ13.2 expressing sub-population was clonal, hereafter referred to as M314.132. This clone was TCRαβ CD4^low^CD8^high^ T cells and expressed a CD8αβ co-receptor.

**Figure 2:** DP T cell clone selection and characterization. A/. Distribution of CD3^+^ T cells subsets based on CD4, CD8 in the M314 ILNL population. Lymphocytes were analyzed after in vitro expansion by three-color flow cytometry using antibodies specific for CD3, CD4 and CD8α or CD8β. Percentage of Vβ13.2 TCR expressing cells was examined on gated the 14% of DP T cells. The Vβ13.2 TCR expressing cells DP T cells were then sorted by FACS. B and C/ TNF secretion by the M314.132 DP T cell clone in response to the autologous melanoma cell line. 10^4^ DP T cells were added to 3×10^4^ M314 melanoma cells in the presence or not of blocking antibodies directed against class I (W6/32), B/C/A24 (B1.23.2), class II (206) HLA and against CD4 and CD8 molecules at the indicated dilutions or concentrations. DP T cell clone reactivity was assessed by a TNF release assay. D/ Time course of CD3 (white) and TCR (black) down-regulation in M314.132 DP T cell clone stimulated with autologous melanoma cell line.

The recognition of the autologous melanoma cell line by M314.132 was inhibited by addition of W6/32 and B1.23.2 Abs, showing that it occurs in the HLA class I context -B, -C or -A24 (Figure 2B). As illustrated by Figure 2C, this recognition was dramatically reduced in the presence of a blocking anti-CD8 antibody, showing that this DP T cell clone was extremely CD8-dependent but not at all CD4-dependent. Furthermore, TCR/CD3 down-modulation induced after autologous melanoma stimulation was observed confirming the implication of this complex in DP T cell clone activation (Figure 2D).

We next performed an extensive phenotypic and functional analysis of the M314.132 clone. The clone was analyzed for the production of a panel of cytokines after stimulation with autologous melanoma cells. As shown in Figure 3A, the clone produce high levels of IL-13, IL-4, TNF-α, GM-CSF, IL-2 and to a lower extent IFN-γ and IL-5. On the other hand, the clone does not synthesize the suppressive cytokines IL-10 and TGF-β (Figure 3A and data not shown). As illustrated by Figure 3B, the clone M314.132 killed the M314 autologous melanoma cell line but not the M132 allogeneic cell line used as negative control (no common HLA with the patient). This lytic activity remains relatively weak as shown by the percentage of lysis not exceeding 20% at an effector/target ratio of 50/1.

**Figure 3:** Functional properties of the M314.132 DP T cell clone. A/ Cytokine production analysis. DP T cell clone was fixed, permeabilized and stained for cytokines following autologous melanoma stimulation. Data are expressed as mean % of intracellular cytokine secreting cells. Open histograms correspond to the analysis of cytokine production by unstimulated M314.132 DP T cell clone (negative control). B/Lysis of the M314 autologous melanoma cell line (closed circles) by M314.132 DP T cell clone. The M132 cell line was used as negative control target (open circles). 51Cr-labeled tumor cells were co-cultured with T cells at various E/T ratios. Chromium release in the supernantants was measured after a 4-h incubation period. C/ Phenotypic characterization of M314 DP T cell clone. D/ Proliferation capacity. CFSE-labeled T cell clones were stimulated with anti-CD3 (OKT3). The CD8 T cell clone used as positive control was obtained by limiting dilution of melanoma specific CD8 T cells. As negative control, T cell clones were maintained in the absence of any stimulation (Not Stimulated: NS).

The DP T cell clone M314.132 expressed high levels of CD45RO and lacked CD45RA, CD27, CD28, CD57and CD62L suggesting the effector/memory phenotype of these cells (Figure 3C).

We therefore analyzed the proliferative response of M314.132 to immobilized anti-CD3 mAbs. As shown in Figure 3D, infiltrating melanoma DP T cell clone exhibited a very poor proliferative response whereas CD8 SP T cell clone, used as positive control, proliferated vigorously in response to the same stimuli. The single positive CD8 T cell clone's proliferation was representative of those of all melanoma infiltrating CD8 T cells. In addition to the lack of proliferation of this DP T cell clone in response to CD3 activation, we failed to expand this clone using the culture protocol used in our laboratory to expand single positive CD8 (or CD4) T cell clones. We investigated, but so far vainly, culture conditions to stimulate optimal proliferation of this DP T cell clone by adding various combinations of cytokines on top of IL-2 (IL-4, IL-7, IL-15 and IL-21) (data not shown). Finally, the only method which let us to obtain a sufficient number of DP clonal cells was a polyclonal expansion of infiltrating M314 lymph node lymphocytes followed by a FACS sorting of Vβ13.2 positive cells corresponding to the M314.132 DP T cell clone.

### HLA-A*2402 Restriction and Recognition of Various Tumors by DP T Cell Clone

To precisely define the HLA restriction and to establish the distribution of the target antigen, we tested M314.132 reactivity towards various tumor cell lines, including melanomas, colon carcinomas, breast carcinomas, renal carcinomas, ovarian carcinomas, lung carcinomas and myelomas, using a TNF-release assay. As shown in Figures 4A and B, this clone recognized all of the melanoma and other tumor cell lines tested expressing the HLA-A*2402 molecule. All tumor cell lines which are not recognized by the DP T cell clone do not express the HLA-A*2402 and/or 2301 molecules. Nevertheless, the production of TNF is lower upon stimulation by the tumor cell lines other than melanomas. This result was in accordance with the inhibition of tumor reactivity observed with B1.23.2 antibody cross-reacting against the HLA-A*2402 (Fig. 2B). In addition, the M314.132 DP T cell clone recognized tumor cell lines expressing the closest matched allele HLA-A*A2301. To complete this study, we transfected a large panel of tumor cell lines by HLA-A*2402 coding cDNA, comprising a variety of cell types as melanomas, breast carcinomas, renal carcinomas, ovarian carcinoma, myeloma and glioblastomas (Figure 4C). All the cell lines transfected with the HLA-A*2402 were recognized according to the transfection's efficiency evaluated by GFP transfection control (data not shown). These data lend support to the recognition by the DP T cell clone M314.132 of a common antigen presented on HLA-A*2402/2301 by cancer cells of different histological origins.

**Figure 4:** Reactivity of M314.132 DP T cell clone against tumor cell lines. A and B/ TNF secretion by the M314.132 DP T cell clone in response to tumor cell lines. 10^4^ DP T cells were added to 3×10^4^ M314 melanoma cells (A) or other tumor cells (B). All tumor cell lines which are not recognized by the DP clone do not express the HLA-A*2402 and/or 2301 molecules. C/ TNF secretion by the M314.132 DP T cell clone to HLA-A*2402 transfected tumor cells. Melanoma (n = 10), breast carcinoma (n = 2), renal carcinoma (n = 1), ovarian carcinoma (n = 1), myeloma (n = 1), and glioblastoma (n = 3) cell lines were transiently transfected with 100ng of HLA-A*2402 plasmid with a lipofectamine reagent kit. 10^4^ DP T cells were added to 3×10^4^ target cells, and the DP T cell clone reactivity was assessed by a TNF release assay. Results are expressed as relative reactivity to the indicated cells in comparison with TNF secretion (100%) induced by M314 autologous melanoma cells.

### Recognition of Various Normal Cells Except Lymphocytes by DP T Cell Clone

To address the question of tumor antigen specificity, we tested the recognition of normal cells from various types. First, M314.132 DP T cell clone recognized HLA-A*2402 positive melanocytes (Mela1) but none of the two non-HLA-A*2402 melanocytes (Figure 5A). However, this reactivity was much lower than that observed against melanoma cell lines. Moreover, diverse normal cell lines including human adipocytes, fibroblasts and embryonic kidney cells as well as african green monkey kidney cells were recognized after HLA-A*2402 transfection (Figure 5B). Nonetheless, the six EBV-B cell lines tested were not recognized by M314 DP T cell clone even the three HLA-A*2402 homozygous cell lines. As EBV-transformed B cell lines have been shown to express the immunoproteasome constituvely [17], we reasoned that if the lack of recognition of homozygous HLA-A*2402 EBV-B cell lines by DP T cell clone was due to their constitutive expression of immunoproteasome, then tumor cells should also lose expression of the epitope after prolonged treatment with IFN-γ. M314 autologous melanoma cell line was treated with IFN-γ for 15 days before being tested for recognition by the clone. As shown in Figure 5D, we observed an inhibition of DP T cell clone recognition. Two CD8 T cell clones were used as controls, one specific for the MELAN-A_26–35_ epitope which is not processed by immunoproteasome and one specific for the MELOE-1_36–44_ epitope which is processed by both standard proteasome and immunoproteasome.

**Figure 5:** Reactivity of M314.132 DP T cell clone against normal cell lines. A/ TNF secretion by the M314.132 DP T cell clone in response to melanocytes. 10^4^ DP T cells were added to 3×10^4^ HLA-A*2402 positive or negative melanocytes, and the clone reactivity was assessed by a TNF release assy. B/ TNF secretion by the M314.132 DP T cell clone to HLA-A*2402 transfected (+) or non-transfected (−) normal cells of different origins and/or species. Results are expressed as relative reactivity to the indicated cells in comparison with TNF secretion (100%) induced by M314 autologous melanoma cells. C/ Lack of recognition of HLA-A*2402 EBV-B lymphocytes. DP T cell clone was fixed, permeabilized and stained for cytokines following stimulation with EBV-B cell lines expressing or not HLA-A*2402 molecules. Data are expressed as mean % of intracellular TNF-α secreting cells. D/ TNF response of DP T cell clone toward melanoma cells treated with or without IFN-γ. Melanoma cells were cultured in the presence or absence of 100U/ml rIFN-γ for 15 days. DP T cell clone and two CD8 T cell clones used as controls were fixed, permeabilized and stained for TNF following stimulation with untreated (white bars) or IFN-γ-treated (hatched bars) melanoma cells. Data are expressed as mean % of intracellular TNF-α secreting cells.

Overall, the M314.132 clone seems to recognize a ubiquitous self antigen processed by the standard proteasome and presented in association with HLA-A*2402/2301 on normal and tumor cells from different species.

## Discussion

The current report provides for the first time functional evidence of tumor reactivity of CD4^+^CD8^+^ DP Tαβ cells in human melanomas. We first observed statistically enhanced frequencies of DP T cells compared to metastasis melanomas (P<0.05) and in invaded lymph nodes (P<0.01) than in normal or patients blood. So, as we previously documented in breast cancer patients [10], this increase of DP T cells is associated with tumor microenvironment. Others studies also reported an increased number of DP T cells in lymphomas [16] and in other diseased individuals [18]–[20].

Of interest, the presence of DP T cells in the target organ of several auto-immune conditions reinforces their involvement in pathologically relevant events. Yet, in humans, very little is known about their antigen specificity and their function. CMV and HIV-1 viral antigen-specific cytotoxic and proliferation responses of DP cells have been observed demonstrating their effector status [21]–[23]. In tumors, there is only one report showing that DP T cells infiltrating a cutaneous T cell lymphoma exert a tumor-specific MHC class-I restricted lysis [15]. Interestingly, our study showed that about 15% of polyclonal melanoma infiltrating DP T cells produce TNF-α in response to autologous tumor cells, demonstrating the frequent anti-tumor reactivity of this new sub-population. This percentage was higher than those observed with SP CD8 suggesting their physiological relevance in tumors.

To further study the phenotype and the function of tumor infiltrating DP T lymphocytes, we isolated a DP T cell clone from invaded lymph node of melanoma patient M314, in which these sub-population represents about 14% of TIL. This DP Tαβ cell clone namely M314.132, co-expressed the CD4^lo^ and the CD8^hi^αβ receptors and displayed an effector memory phenotype. M314.132 DP T cell clone recognized autologous melanoma cells in MHC class I restricted context with a very strong CD8 dependence. In response to autologous melanoma cell line, this clone is lytic and produced in decreasing order the following Th1 and Th2 cytokines: IL-13, IL-4, TNF-α, GM-CSF, IL-2, IFN-γ and IL-5. This original cytokinic profile was also observed on polyclonal melanoma infiltrating DP T cells in response to CD3 stimulation and was similar on polyclonal breast tumor associated DP T cells as we previously reported [10]. In comparison to SP T cells, DP T cells have much greater capacity to produce Th2 cytokines, especially regulatory cytokines such as IL-13 (75% of cytokines secreting cells), IL-4 (40%) and IL-5 (21%). Terabe and Berzofsky single out IL-13, produced by type II NKT cell in several mouse tumor models, as an important immunosuppressive cytokine, inducing CD11b^+^Gr-1^+^ myeloid lineage to secrete TGF-β that finally inhibits CTL induction against the tumor [8], [24], [25]. It has also been reported that human CD4^+^ regulatory NKT cells can suppress the expansion of tumor antigen-specific CTLs via Th2 cytokines such as IL-4 and IL-10 [26]. In addition, it has been documented that IL-13 and IL-4 downregulated arginase production in melanomas, leading to down-regulation of CD3ζ expression thus limiting T cell function [27]. In contrast, another study reported that the massive production of IL-4 and IL-13 by the CD4 subset of invariant NKT, together with IFN-γ, induced IL-12 production by the dendritic cells leading to a shift toward Th1 responses [8], [28]. The last cytokine specifically produced by DP T cells, IL-5, is generally regarded as a Th2 cytokine involved in eosinophil maturation and function and in B cell growth and antibody production. However, Apostolopoulos and collaborators have demonstrated *in vivo* in a mouse model the role of IL-5 in the generation of a functional cytotoxic response to tumors [29]. Moreover, high amounts of IL-5 have been shown to be produced by a fraction of human CD4^+^ invariant NKT [30]. Therefore, considering their cytokinic profile, it is conceivable that melanoma infiltrating DP T cells might play, at the effector level, roles similar to those of regulatory invariant NKT.

One major difference between SP T cells and DP T cells *in vitro* is the limited capacity to divide displayed by DP T cells. This poor proliferative capacity could be due to short TREC (T cell Receptor Excision Circles) levels. Indeed, it has been reported that DP T cells displayed lower TREC content than SP cells, demonstrating at the molecular level that DP T cells experienced more cells divisions than their SP counterparts [21].

With regard to antigen specificity of DP T cells, we show that M314.132 clone, which was restricted by HLA-A*2402 (and the very similar HLA-A*2301 allele), recognized both tumor and normal cells from different origins. We speculated that the target antigen could be a ubiquitous self-antigen. The recognition of ubiquitous self antigens by tumor infiltrating CD8 T lymphocytes has already been described in renal and prostate cancers [31], [32]. On account of their abundant and ubiquitous nature, these antigens may represent a new type of tumor-associated antigens. Hypothetically, these antigens would be derived from ubiquitously expressed proteins that, under normal circumstances, are not efficiently processed. However, despite the probable expression of ubiquitous antigens, homozygous HLA-A*2402 EBV-B cells were not recognized by the DP T cell clone. In addition, we observed an inhibition of DP T cell clone recognition of IFN-γ long-pretreated autologous melanoma cells, which could be attributed to the replacement of the standard proteasome by the immunoproteasome. This observation additionally supports our hypothesis that although EBV-B cells express ubiquitous self Ags, they are not capable of processing the epitope recognized by the DP T cells due to their constitutive expression of immunoproteasome. A major difference between the two forms of proteasomes in terms of catalytic activity is the severely reduced ability of the immunoproteasome to cleave after acidic residues and after residues with branched side chains [33]–[35]. This last point could explain why Melan-A as RU1, gp100 and tyrosinase epitopes having a valine at their C terminus are not cleaved by the immunoproteasome [31], [36]. This could also be the case for HLA-A*2402 epitopes for which branched amino acids as leucin or isoleucin have been reported among their predictable anchor sites. The notion that the immunoproteasome is more competent at producing class-I-binding peptides probably remains true for many epitopes. However a number of epitopes, mainly derived from self proteins, are not processed efficiently by the immunoproteasome. This provides a plausible explanation for DP T cells escape negative selection in the thymus where a high level of immunoproteasome has been observed [37]. It could also explain why such cells did not undergo autoimmune activation, again because mature dendritic cells, which are considered as the major antigen-presenting cells capable of activating naive T cells, only carry immunoproteasomes [38].

Concerning the origin of DP T cells, several studies hypothesized that they could derive from SP cells. It has been demonstrated that IL-4 represents an important soluble mediator of CD8αα induction on human SP CD4 T cells [39]. On the other hand, when activated *in vitro* via TCR cross-linking, SP CD8αβ T cells may become capable of expressing low levels of CD4 [40]. Nevertheless, M314.132 clone as well as polyclonal DP T cells were found to express high levels of both CD4 and CD8αβ molecules during all time of culture, ruling out the hypothesis of the acquisition of a second CD4 or CD8 co-receptor. Moreover, the M314.132 DP T cell clone, representing more than 60% of the M314 DP T cell subset expressed the Vβ13.2, which is not used by the M314 SP T cell subsets (data not shown). Therefore, as judged by their TCR Vβ usage, and in accordance with earlier studies on DP T cells present in lesional skin of patients with systemic sclerosis, melanoma infiltrating DP T cells would have a clonal origin distinct from that of SP CD4^+^ and CD8^+^ SP cells [13].

Another question concerns the increase of the frequencies of DP T cells in some tumors. In previous studies, the higher expression of CXCR3 and CCR6 chemokines receptors on DP T cells compared to SP T cells have been described that could explain their recruitment in tumors [12], [41]. Nonetheless, we observed that M314.132 DP T cell clone express poorly CCR6 and not at all CXCR3 (data not shown). The molecules and cytokines involved in the recruitment and/or propagation of DP T cells in melanomas have to be clearly identified.

In conclusion, although the function of this DP T cell population remains to be defined *in vivo*, we can postulate that, according to their broad tumor reactivity and to their cytokinic potential, these cells could participate in immune responses to tumors. The clinically relevant function of these tumor associated DP T cells needs to be carefully analyzed in order to develop appropriate immunotherapeutic strategies.

## Materials and Methods

### Antibodies

The phenotype of cells was analyzed using monoclonal antibodies (mAbs) in conjunction with three or four color immunofluorescence. The mAbs used in this study include fluorescein isothiocyanate (FITC)-, phycoerythrin (PE)-, allophycocyanin (APC)-, peridin-chlorophyll-protein complex (PerCp)-conjugated reagents against CD3, CD4, CD27, CD28, CD45-RA, CD45-RO, CD57, CD62-L, IL-2, IL-4, IL-5, IL-13, TNF-α, IFN-γ, GM-CSF from BD Biosciences, CD8α, CD8β, TCRαβ, Vβ1, -2, -3, -4, -5.1, -5.2, -5.3, -7, -7.2, -8, -9, -11, -12, -13.1, -13.2, -13.6, -14, -16, -17, -18, -20, -21.3, -22, and -23, from Beckman Coulter. mAbs used for blocking experiments against HLA class I (clone W6.32), HLA-B/C (clone B1.23.2), HLA class II (clone 206) were produced in our laboratory from hybridomas obtained from the American Type Culture Collection for W6.32 Ab and from F. Lemonier (Pasteur Institute, Paris, France) for B1.23.2 Ab.

### Patients and Specimens

Peripheral blood (n = 6), metastasis (n = 10), invaded lymph nodes (n = 30) were collected from patients with melanoma and peripheral blood (n = 11) from healthy donors, all with formal consent.

### Ethics Statement

Written consents were obtained from all patients and healthy donors. All these studies were approved by the local ethics committee “Comité de Protection des Personnes Ouest IV-Nantes” and the “Agence française de sécurité sanitaire des produits de santé”.

### Isolation of Polyclonal Cell Populations (TIL, ILNL and PBMC)

Solid tumor fragments of primary tumor or tumor invaded lymph node were mechanically disaggregated. Tumor Infiltrating Lymphocytes (TIL) and tumor Invaded Lymph Node Lymphocytes (ILNL) were isolated by culturing disaggregated tumor fragments into 24-well tissue culture plates with RPMI 1640 (Sigma-Aldrich) containing 8% human serum (local production), 100U/mL penicillin, 100µg/mL streptomycin (Sigma-Aldrich), 2mM L-glutamine (Sigma-Aldrich) and 150U/ml rIL-2 (Eurocetus, Rueil-Malmaison, France) for 10–14 days. These populations were then expanded by a single round of stimulation with PHA-L (Sigma-Aldrich) in the presence of irradiated feeder cells (allogeneic lymphocytes and B-EBV B cells), as described [42], [43]. The expanded lymphocytes were transferred into 6-well tissue culture plates with fresh medium to maintain a cell density of 0.5 to 1.5×10^6^ cell/mL.

PBMC (Peripheral Blood Mononuclear Cells) were isolated from blood by a Ficoll density gradient (Eurobio, Les Ulis, France).

### Sorting DP T Cell Clone M314.132 with Facs Aria

First, polyclonal lymphocytes from M314 patient were labeling with Vβ13.2 mAb following a standard cell surface staining procedure. The sorting was performed on a Facs Aria (Becton Dickinson, Grenoble, France). Gates were set up to exclude nonviable cells and debris. Sorted DP T cell clone was assessed to ensure its purity.

### Cell Lines Culture

Melanoma cells lines, colorectal carcinoma cell line C4-A and renal carcinoma cell lines (R3 and R9) were established, respectively, in the GMP Unit of Cellular Therapy and in our laboratory. Mouse fibrosarcoma WEHI 164 clone 13 (established by M. Rollinghoff and N.L. Warner) and COS-7 cells (established by Y. Gluzman) were obtained from T. Boon (Ludwig Institute for Cancer Research, Brussels, Belgium). Ovary carcinoma cell line (OVCAR-3) (established by T.C. Hamilton), renal carcinoma cell line (A498) (established by D.J. Giard) and non-small cell lung cancer cell line (1355) (established by H. Oie) were gifts from C. Saï (UMR 892 INSERM/Université de Nantes, France). Colorectal carcinoma cell lines, LS174T and LS180 (established by B.H. Tom), SW480 (established by J. Fogh), SW707 (obtained from the DKFZ tumor bank), SW1116 (established by W.C. Wright), glioblastoma cells lines, U-251 (established by D.D. Bigner), GBMS1 and GBS (established by M. Gregoire), and HFF-2 fibroblast cell line (established by ATCC) were gifts from M. Grégoire (UMR 892 INSERM/Université de Nantes, France). Myeloma cells lines, XG-7 (established by X.G. Zhang), KMM1 (established by Dr Otsuki), NCI-H929 (established by G.F. Hollis), OPM-2 (established by Dr Katagiri), LP1 (established by Dr Pegoraro) were gifts from C. Pellat (UMR 892 INSERM/Université de Nantes, France). Breast cancer cell lines, CAMA-1 (established by J. Fogh), MDAMB-231 and MDAMB-468 (established by R. Cailleau) were gifts from D. Jäger (Klinik und Poliklinik für Onkologie, Zürich, Suisse). Breast cancer cell line S68 was established and gift from V. Catros (UPRES EA, 3891, Rennes, France). Breast cancer cell line MCF-7 (established by B.J. Sugarman), was obtained from the American Type Culture Collection. Normal melanocytes were established and gifts from M. Regnier (L'Oréal Laboratory, Paris, France). EBV-B cell lines were established and gifts from C. Reutière (EFS, Nantes, France). Human adipocytes PAZ-6 (established by V. Zilberfarb) were a gifts from J-P. Segain (UMR 1280 INRA/Université de Nantes, France).

### T Cell Clones

Melanoma-reactive CD8 αβ T cell clones specific for Melan-A/MART-1 (AAGIGILTV) and MELOE-1 (TLNDECWPA) epitopes were derived in our laboratory either from TIL or from peptide stimulated PBMC.

### Immunofluorescence Analysis

Two ×10^5^ cells were stained with isotype controls or with one or four antibodies for 20 minutes at 4°C. Cells were then washed and 10^5^ cells were acquired in the viable cells gate on a FACScalibur flow cytometer using Cellquest software (Becton Dickinson, Grenoble, France).

### Transient Transfection of Cell Lines by the HLA-A*2402 cDNA

The HLA-A*2402 cDNA was cloned from the M314 melanoma cell line. Cells were seeded in 96-well plates and incubated until they were 80% confluent. The expression plasmid carring the HLA-A*2402 cDNA (100ng) was mixed for 30 minutes with Reagent Plus (1µl), Lipofectamine Reagent (0.5µl) in 20µl of Optimem I medium (Life Technologies). Cells were washed by replacing the complete medium by the Optimem I medium (50µl). Then, the HLA-A*2402/Lipofectamine mix was added in each well. After 3 hours of incubation, complete medium (130µl) was added to the transfection mixture.

### Analysis of TNF Production

Measurement of TNF produced by T cells in response to tumor cells or transfected tumor cells was performed as previously described, using WEHI 164 clone 13 cells [44]. For blocking experiments, melanoma cell lines or DP T cell clone were pre-incubated with different Abs.

### Analysis of Intracellular Cytokines by Flow Cytometry

Lymphocytes were stimulated by OKT3 (5µg/mL, Clinisciences) or tumor cells, in 200µl of RPMI 1640-10% FCS in the presence of Brefeldin A, 10µg/ml (Sigma, St Louis MO, USA) for cytokine analysis in round-bottom 96-well plates. The cultures were incubated for 6 hours at 37°C in 5% CO_2_ humidified atmosphere. Cells were then stained at 4°C for 20 minutes, with anti-CD4 and anti-CD8 Abs for extracellular staining. For intracytoplasmic staining, cells were washed two times in 0.1% PBS BSA, fixed 10 minutes at room temperature in a solution of PBS 4% paraformaldehyde (Sigma), washed again and stored at 4°C until labeling. Specific mAbs (cytokines) were added to fixed cells and incubated for 30 minutes at room temperature. Reagent dilutions and washes were made with PBS containing 0.1% BSA and 0.1% saponin (Sigma). After staining, cells were resuspended in PBS and 10^5^ viable cells were acquired on a FACScalibur cytometer using Cellquest software. According to the FSC/SSC parameters, lymphocytes were gated and the autologous melanoma cells were excluded. using Cell Quest Pro software.

### Analysis of Lytic Activity

Cytotoxic activity of T cells was measured in a standard 4-h assay against ^51^Cr-labeled cells. Briefly, tumor cell lines were labeled with 100µCi Na^51^CrO_4_ (Oris Industrie, Gif-sur-Yvette, France) for 1h at 37°C, and incubated, 4h at 37°C, with effectors T cells at various ratios. The radioactivity, released by target cells, was measured on a beta plate counter (EG&G Wallac, Evry, France).

### CD3 and TCRαβ Downregulation

CD3 or TCRαβ fluorescence intensity was measuring in unstimulated and activated lymphocytes with tumor cells following a standard cell surface staining procedure. Data were expressed as percentages of cells showing a CD3 and TCRαβ downregulation.

### Proliferation Assay

Lymphocytes were labeled with CFSE (Sigma-Aldrich) as described previously [45]. The 5 mM stock solution of CFSE in DMSO (Sigma-Aldrich) was diluted to 5 µM in a volume of PBS equal to that in which cells (1×10^7^ cells/ml in PBS) were suspended, and the cells were then incubated at 37°C for 10 min. The labeling process was quenched by adding an equal volume of heat-inactivated FBS (Invitrogen) to the sample. After 1 min, CFSE-labeled cells were washed three times, recounted, and adjusted to a concentration of 5×10^5^ cells/ml in the culture medium. 10^5^ CFSE-labeled lymphocytes were then incubated with 200µl RPMI 1640-8% SH and 150U/ml rIL-2 in round-bottom 96-well plates in the presence or absence of OKT3 (5µg/mL, Clinisciences). After 5 days, cells were suspended in PBS/BSA and tested for fluorescence using a Becton Dickinson FACSCalibur with CellQuest™ Pro. FACS data and CFSE intensity were analyzed using FlowJo (version 7, Tree Star, Inc. Oregon, USA). In this experiment, a single positive CD8 T cell clone, obtained by limiting dilution of melanoma specific CD8 T cells, was used as positive control of proliferation.

### Statistical Analysis

Statistical analysis was done with InStat 2.01. Data were analyzed using Tukey-Kramer multiple comparisons test. P<0.05 was considered significant.
